The article "Moringa leaf extract improves biochemical attributes, yield and grain quality of rice (Oryza sativa L.) under drought stress" was retracted in 2022. Reasons: compromised peer review; a conflict of interest; concerns about the authorship.

# Moringa leaf extract improves biochemical attributes, yield and grain quality of rice (*Oryza sativa* L.) under drought stress

**DOI:** 10.1371/journal.pone.0254452

**Published:** 2021-07-16

**Authors:** Shahbaz Khan, Abdul Basit, Muhammad Bilal Hafeez, Sohail Irshad, Saqib Bashir, Safdar Bashir, Muhammad Mudassar Maqbool, Muhammad Sohail Saddiq, Zuhair Hasnain, Bandar S. Aljuaid, Ahmed M. El-Shehawi, Yunzhou Li

**Affiliations:** 1 Department of Agronomy, Ghazi University, Dera Ghazi Khan, Pakistan; 2 National Agricultural Research Centre, Islamabad, Pakistan; 3 Department of Plant Pathology, College of Agriculture, Guizhou University, Guiyang, Guizhou, China; 4 Department of Agronomy, Northwest A & F University, Yangling, Xianyang, China; 5 In-Service Agricultural Training Institute, Rahim Yar Khan, Pakistan; 6 Department of Soil & Environmental Science, Ghazi University, Dera Ghazi Khan, Pakistan; 7 Pir Mehr Ali Shah Arid Agriculture University, Rawalpindi, Pakistan; 8 Department of Biotechnology, College of Science, Taif University, Taif, Saudi Arabia; Harran Üniversitesi: Harran Universitesi, TURKEY

## Abstract

Changing climate, food shortage, water scarcity and rapidly increasing population are some of the emerging challenges globally. Drought stress is the most devastating threat for agricultural productivity. Natural plant growth substances are intensively used to improve the productivity of crop plants grown under stressed and benign environments. The current study evaluated whether leaf extract of different moringa (*Moringa oleifera* L.) could play a role in improving drought-tolerance of rice (*Oryza sativa* L.). Rice plants were grown under three drought conditions, i.e., no, moderate and severe drought (100, 75 and 50% field capacity, respectively). Moringa leaf extract (MLE) obtained from four landraces (Multan, Faisalabad, D. G. Khan and exotic landrace from India) was applied during critical crop growth stages, i.e., tillering, panicle initiation and grain filling. Drought stress adversely affected the gas exchange attributes, photosynthetic pigments, antioxidant enzymes’ activities, yield and quality parameters of rice. Application of MLE from all landraces significantly improved physiological, biochemical and yield parameters under stressed and normal environmental conditions. The highest improvement in gas exchange traits (photosynthetic rate, stomatal conductance and respiration rate), photosynthetic pigments (chlorophyll *a*, *b* and carotenoids) and enzymatic activities (superoxide dismutase, catalase) and oxidative marker (H_2_O_2_) was recorded with MLE obtained from Faisalabad landrace. The application of MLE of Faisalabad landrace also improved yield and grain quality of rice grown under drought stress as well as drought-free environment. Thus, MLE of Faisalabad can be successfully used to improve growth, productivity and grain quality of rice under drought stress.

The article "Moringa leaf extract improves biochemical attributes, yield and grain quality of rice (Oryza sativa L.) under drought stress" was retracted in 2022. Reasons: compromised peer review; a conflict of interest; concerns about the authorship.

## Introduction

Changing climate, food shortage, water scarcity and rapidly increasing population are some of emerging challenges globally faced by the agricultural community. Drought stress is the most devastating threat for agricultural productivity [1]. Globally, rice (*Oryza sativa* L.) was grown on 167 million hectares (M ha) and ranked third highest cereal in terms of production [495.87 million tones (MT)] following maize (*Zea mays* L.) and wheat (*Triticum aestivum* L.) during 2019 [2]. Rice serves as a staple food for >3 billion people and provides 20% of world’s dietary energy supply, while wheat and maize supply 19 and 5%, respectively. Drought stress is a main limiting factor for crops produced in rain fed areas of Asia, affecting >23 M ha of land. Drought stress reduces photosynthetic pigments, CO_2_ intake, photosynthesis and relative water contents, impairs cell division and elongation [3] and disturbs the balance between reactive oxygen species (ROS) and antioxidants [4]. Roots of rice seedling are also very sensitive to abiotic stresses because they inhibit the cell expansion and other attributes of root development system [5]. Nevertheless, enzymatic antioxidants such as superoxide dismutase (SOD), peroxidase (POD) and catalase (CAT), and non-enzymatic antioxidants play a vital role in detoxifying ROS [6]. Drought stress is very harmful at reproductive and grain-filling stages as it affects pollination, causes male sterility and decreases grain formation in rice. Drought stress also decreases grain-filling rate and duration, grain weight and grain yield [7].

Accumulation of compatible solutes, reduced stomatal conductance and activation of antioxidant defense systems are important mechanisms help plants withstand drought stress [8]. Various approaches could be used to mitigate the adverse effects of drought stress, including use of drought-tolerant cultivars, natural and synthetic mulches, stress-signaling molecules, osmo-protectants and crop/plant water extracts. Being biologically safe and economically sustainable, crop/plant water extracts have a great potential for crop enhancement under stressful environments in recent years [9]. Water extracts of various parts of agronomic crops have been identified which improved the growth and development of plants under normal as well as stressful environments through modulating phytohormones metabolism, photosynthesis, antioxidant defense system, stomatal conductance, water/nutrient absorption, signal transduction, gene expression, leaf senescence and grain partitioning [10]. Water extract of prickly chaff flower (*Achyranthes aspera* L.), a broadleaf annual herbaceous plant, is also being used in the agriculture because it has allelopathic potential [11]. Application of biostimulant particularly humic acid in combination with micronutrients (B, Zn) significantly improved the growth, grain-filling rate and yield attributes of wheat crop [12].

The article "Moringa leaf extract improves biochemical attributes, yield and grain quality of rice (Oryza sativa L.) under drought stress" was retracted in 2022. Reasons: compromised peer review; a conflict of interest; concerns about the authorship.

Moringa (*Moringa oliefera* L.) has received significant attention among the scientific community because it is a rich source of mineral nutrients, growth hormones, vitamins and antioxidants in leaves [9, 13]. It is a potential allelopathic crop and its CWE are used due to the presence of several allelochemicals [14, 15]. Application of moringa leaf extract (MLE) to plant foliage has been reported to boost seedling establishment, plant growth and ultimately yield of field crops cultivated under normal and stressful environments [9, 16, 17]. Therefore, the current study investigated potential of leaf extracts obtained from local and exotic moringa landraces in improving growth, biochemical attributes, yield and grain quality of rice cultivated under normal and drought stressed environments. The results of the study will help to improve rice productivity under drought stressed environments.

## Materials and methods

### Experimental particulars

This study was conducted during the rice growing season 2019 to explore the impact of moringa leaf extracts obtained from local and exotic landraces on emergence, growth, yield and quality parameters of rice (cv. Basmati Pak) grown under drought stressed and drought-free environments. The experiment was laid out according to completely randomized design with split plot arrangements. The experiment was conducted in wire-house at Department of Agronomy, Ghazi University, Dera Ghazi Khan (30.05° N, 70.64° E and 129 m asl), Pakistan. Earthen pots (45 cm in height and 30 cm in diameter) were filled with growth media. Growth media consisted of compost, sand, silt and clay with equal proportion. The growth media had sand (44.19%), clay (20.29%) and silt (35.52%) with pH and EC of 7.7 and 2.59 dS m^-1^, respectively. Rice seeds were purchased from Punjab Seed Corporation, Faisalabad-Pakistan. Ten seeds were sown in each pot. After 15 days of emergence, thinning was done and only four seedlings were maintained in each pot.

### Drought stress treatments, extract preparation and application

Three different drought stress levels, i.e., control (CC) where pots were maintained at 100% field capacity, moderate drought stress (MDS) where pots were maintained at 75% field capacity and severe drought stress (SDS) in which pots were maintained at 50% field capacity. The MLE treatments included water spray (WS), foliar application MLE obtained from Multan landrace (MLE-LM), foliar application MLE Faisalabad landrace (MLE-LF), foliar application MLE D. G. Khan landrace (MLE-LD) and foliar application MLE obtained from PKM1 exotic landrace (MLE-EL).

The article "Moringa leaf extract improves biochemical attributes, yield and grain quality of rice (Oryza sativa L.) under drought stress" was retracted in 2022. Reasons: compromised peer review; a conflict of interest; concerns about the authorship.

The drought stress levels (CC, MDS and SDS) were induced by maintaining the pots at respective field capacity by limiting the water supply. The soil moisture contents were maintained throughout the growth period of rice plants starting from transplantation to maturity. In order to determine the water loss by transpiration, pots were weighed daily and transpired amount of water was replenished. The FC was determined according to gravimetric method proposed by Nachabe [18].

Fresh, mature, disease-free and healthy moringa leaves were collected form well-established trees at respective locations, rinsed with tap water and kept in refrigerator overnight. Extraction was done with a locally assembled machine [14]. The extracts were sieved and diluted with distilled water to prepare 3% solution. The MLE in all treatments was sprayed during critical growth stages of rice, i.e., tillering, panicle initiation and grain-filling. A hand shower of one-liter capacity was used for foliar spray. The WS was regarded as a control treatment for comparison with MLE treatments.

### Estimation of gas exchange attributes

Gas exchange attributes were recorded three days after MLE application during grain-filling stage. Flag leaf of rice plants was used for the measurements during 10:00 am to 12:00 pm. Photosynthesis rate (*A*) (μmol CO_2_ m^-2^ s^-1^), stomatal conductance (*gs*) (mmol m^-2^ s^-1^) and respiration rate (E) (mmol H_2_O m^-2^ s^-1^) were estimated according to procedure described by Long [19] using an infrared gas analyzer (IRGA) *LI-6400* portable device. The rate of water loss and rate of CO_2_ uptake are used to assess the rate of transpiration and photosynthetic carbon assimilation, respectively is a working principle of *LI-6400*.

### Physiological attributes

Top leaf samples were collected three days after MLE spray during grain-filling stage to record the chlorophyll *a*, *b* and carotenoids. To measure the chlorophyll *a*, *b* and carotenoid contents, absorbance of filtrate was determined at 663, 645 and 480 nm, respectively according to Arnon [20] by using Spectrophotometer. The following formulas were used to record chlorophyll *a*, *b* and carotenoid contents;

Chlorophylla=[12.7(OD663)−2.69(OD645)×V/1000×W

Chlorophyllb=[12.7(OD645)−4.68(OD663)×V/1000×W

Carotenoids=[(OD480)+0.114(OD663)−0.638(OD645)]×V/1000×W

Here, V = volume of the extract (ml), W = weight of the fresh leaf (g)

Total chlorophyll contents were calculated by adding chlorophyll *a* and *b* contents.

The article "Moringa leaf extract improves biochemical attributes, yield and grain quality of rice (Oryza sativa L.) under drought stress" was retracted in 2022. Reasons: compromised peer review; a conflict of interest; concerns about the authorship.

### Enzymatic attributes

Data regarding enzymatic attributes were recorded three days after MLE spray at grain-filling stage. The SOD activity was measured according to Giannopolotis and Ries [21]. The activity of CAT was recorded by using spectrophotometer with the performance set according to Chance and Maehly [22]. Ascorbate peroxidase (APX) activity was estimated according to Nakano and Asada [23] with slight modification. The H_2_O_2_ was measured by following the procedure of Velikova [24].

### Agronomic and yield-related traits

Plant height was measured at maturity using a meter rod. Total numbers of productive tillers per plant were counted from each replication and averaged. Panicle length was measured with the help of scale from five randomly selected tillers and averaged. In case of kernels per panicle, five panicles were taken from each treatment, kernels were counted and averaged. The 1000-kernel weight was calculated by counting the 1000 kernels and weighing on an ordinary balance. For the determination of grain yield, fully matured plants were harvest and grains obtained from each treatment after threshing were weighed.

### Quality parameters

The protocol proposed by Zhu [25] was followed to determine the amylopectin and amylose contents rice grains. The collected samples of rice grains were first ground using a mortar and powder was degreased two times with anhydrous ether. A fraction of 100 mg from each sample was used to measure the amylopectin and amylose contents. After drying the samples in an oven, sub-samples were run in Microkjeldahl apparatus to determine total proteins following Latimer [26].

### Statistical analysis

Collected data of growth, yield and quality parameters were analyzed using statistical package “Statistic 8.1”. Fisher’s analysis of variance (ANOVA) technique was used to test the significance in the data. Microsoft Excel was used for calculation of standard errors of means and graphical presentation. The differences among treatment means were assessed using LSD post-hoc test at 5% probability [27].

## Results

Significant levels of gas exchange, physiological, enzymatic, agronomic, yield and quality attributes as affected by drought stress and MLE are presented in Table 1. Impact MLE obtained from local and exotic landraces on *A*, *gs* and *E* under normal and drought stressed environments is presented in Fig 1. Physiological parameters like *A*, *gs* and *E* significantly varied under different drought stress treatments. The highest *A*, *gs* and *E* were observed maximum under CC followed by MDS, while SDS recorded the lowest values of these physiological parameters. The MLE obtained from all landraces significantly influenced *A*, *gs* and *E* compared to control. The highest *A* was recorded for MLE-LF, which was similar to MLE-LD and MLE-LM. The highest *gs* was noted for MLE-LF followed by MLE-LD and MLE-LM. The MLE-LF recorded the highest *E* followed by MLE-LM, MLE-LD and MLE-EL (Fig 1A–1C).

The article "Moringa leaf extract improves biochemical attributes, yield and grain quality of rice (Oryza sativa L.) under drought stress" was retracted in 2022. Reasons: compromised peer review; a conflict of interest; concerns about the authorship.

**Fig 1:** Impact of leaf extracts from local and exotic moringa landraces on photosynthesis rate (*A*) (a), stomatal conductance to water (*gs*) (b) and respiration rate (*E*) of rice cultivated under normal and drought-stressed environments (n = 4).

**Table 1:** Analysis of variance for gas exchange, physiological, enzymatic, agronomic, yield and quality attributes of rice plants cultivated under different levels of drought stress and foliar application of moringa leaf extract (n = 4).

SOV	DF	*A*	*gs*	*E*	Chlo *a*	Chlo *b*	Total Chlo	Carotenoids	SOD	CAT	APX
WT	2	206.8**	73.98*	0.152*	21.03*	3.865*	42.93*	1.716*	83.65*	1.841*	1.274*
FT	4	2.264*	3.294*	0.002*	0.881*	0.162*	1.801*	0.072*	42.64*	10.58*	7.272*
WT×FT	8	0.030^NS^	0.018^NS^	0.001^NS^	0.016*	0.003*	0.034*	0.001*	7.462*	1.981*	1.603*
SOV	DF	H_2_O_2_	Plant height	Tillers per plant	Panicle length	Kernels per panicle	1000-kernel weight	Grain yield	Amylose	Amylopectin	Protein
WT	2	499.3**	4278*	32.62*	87.68*	7009*	265.1**	10156*	184.6*	184.6**	87.13**
FT	4	35.32*	183.9*	25.69*	42.27*	234.6*	21.59*	311.8*	8.415*	8.415*	0.079^NS^
WT×FT	8	6.612*	1.101^NS^	0.617^NS^	1.074^NS^	4.401^NS^	1.537*	25.20^NS^	0.479^NS^	0.479^NS^	0.072^NS^

SOV = source of variance, WT = water treatments, FT = foliar treatments, WT × FT = interaction of water and foliar treatments, DF = degree of freedom, *A* = photosynthesis rate, *gs* = stomatal conductance to water, *E* = respiration rate, Chlo = chlorophyll, SOD = superoxide dismutase, CAT = catalase, APX = ascorbate peroxidase,

* = significant at P < 0.05,

** = significant at P < 0.01.

The impact MLE treatments on chlorophyll *a* & *b*, total chlorophyll and carotenoids is presented in Fig 2A–2D. The chlorophyll *a*, *b*, total chlorophyll contents and carotenoids significantly differed under various drought stress levels. Moreover, MLE of various landraces significantly influenced biochemical parameters. Interactive effect of drought stress and MLE was also significant. The highest chlorophyll *a*, *b*, total chlorophyll contents and carotenoids were recorded for CC with MLE-LF, while the lowest values of these parameters were recorded under SDS with WS. The MLE from all landraces resulted in better biochemical parameters than control. The MLE from all landraces improved biochemical parameters under MDS and SDS (Fig 2A–2D).

The article "Moringa leaf extract improves biochemical attributes, yield and grain quality of rice (Oryza sativa L.) under drought stress" was retracted in 2022. Reasons: compromised peer review; a conflict of interest; concerns about the authorship.

**Fig 2:** Impact of leaf extracts from local and exotic moringa landraces on chlorophyll *a* (a), chlorophyll *b* (b), total chlorophyll (c) and carotenoid contents (d) of rice leaf cultivated under normal and drought-stressed environments (n = 4).

Impact of MLE on enzymatic activities and H_2_O_2_ under different drought stress treatments is presented in Fig 3. The severe drought stress with MLE-LF had the highest activity of superoxide dismutase, which was statistically similar to leaf extracts of local and exotic landraces. The lowest activity of superoxide dismutase was observed under control conditions with water spray. The catalase and ascorbate peroxidase activities significantly varied under different drought stress levels with foliar treatments. The severe drought stress with MLE-LF recorded the highest activities of catalase and ascorbate peroxidase, while the lowest activities were noted under severe drought stress with water spray. The severe drought stress with water spray had the highest H_2_O_2_ contents, while remaining MLE treatments under control conditions recorded the lowest H_2_O_2_ production (Fig 3A–3D).

**Fig 3:** Impact of leaf extracts from local and exotic moringa landraces on superoxide dismutase (SOD) (a), catalase (CAT) (b), ascorbate peroxidase (APX) (c) and hydrogen peroxide (H_2_O_2_) (d) of rice leaf cultivated under normal and drought-stressed environments (n = 4).

Data regarding plant height is presented in Table 2. The MLE-LF significantly improved plant height followed by MLE-LD and MLE-LM, while the lowest was noted for WS. The longest plants were recorded for CC followed by MDS, while SDS produced the shortest plants. The highest number of productive tillers per plant were observed under CC, while SDS resulted in the lowest number of productive tillers per plant. The MLE obtained from all landraces improved number of productive tillers per plant compared to WS; however, MLE-LF produced the highest number of productive tillers per plant followed by MLE-LD, MLE-LD and MLE-EL, respectively (Table 2). Panicle length significantly varied under different drought stress levels. The CC observed the longest panicle length followed by MDS, while shortest panicles were observed under SDS. The MLE-LF significantly improved panicle length of rice crop, while the lowest panicle length was recorded under WS (Table 2). The number of kernels per panicle significantly varied under different drought stress treatments. The highest number of kernels per panicle were recorded for CC followed by MDS, the lowest number of kernels per panicle were observed under SDS (Table 3). The MLE-LF significantly improved number of kernels per panicle and WS recorded the lowest number of kernels per panicle (Table 3). Individual and interactive effect of drought stress and MLE treatments significantly altered 1000-kernel weight. The MLE-LF applied under CC recorded the heaviest 1000-kernels, whereas WS under SDS resulted the lightest 100kernels (Table 3). The highest grain yield was noted under CC followed by MDS, while SDS recorded the lowest grain yield. Among MLE originated from different landraces, MLE-LF produced the highest grain yield followed by MLE-LM, MLE-LD and MLE-EL, respectively (Table 3).

The article "Moringa leaf extract improves biochemical attributes, yield and grain quality of rice (Oryza sativa L.) under drought stress" was retracted in 2022. Reasons: compromised peer review; a conflict of interest; concerns about the authorship.

**Table 2:** Impact of leaf extracts from local and exotic moringa landraces on plant height, number of productive tillers and panicle length of rice cultivated under different levels of drought stress (n = 4).

Treatments	Plant height (cm)				Productive tillers per plant				Panicle length (cm)			
	CC	MDS	SDS	Mean (FT)	CC	MDS	SDS	Mean (FT)	CC	MDS	SDS	Mean (FT)
WS	108.25	96.00	79.50	94.58 D	9.00	7.00	6.00	7.33 D	18.25	17.00	15.25	16.83 D
MLE-LM	116.25	102.25	86.75	101.75 B	11.00	10.00	8.30	9.75 BC	22.50	19.75	17.50	19.92 B
MLE-LF	119.00	105.25	90.50	104.92 A	13.00	11.00	10.00	11.33 A	24.50	21.87	19.50	21.96 A
MLE-LD	116.50	102.50	86.13	101.71 B	11.30	9.80	9.30	10.08 B	22.00	19.69	17.25	19.65 B
MLE-EL	112.75	99.00	83.75	98.50 C	10.00	9.50	8.00	9.17 C	20.12	18.75	16.94	18.61 C
Mean (WT)	114.55 A	101.00 B	85.32 C		10.90 A	9.50 B	8.30 C		21.46 A	19.41 B	17.28 C	
LSD, 0.05	WT = 0.8921, FT = 1.2136, WT×FT = NS				WT = 1.0171, FT = 0.6516, WT×FT = NS				WT = 1.0036, FT = 0.6623, WT×FT = NS			

Means sharing the same alphabets did not differ significantly at P ≤ 0.05. NS = statistically non-significant, CC = control condition, MDS = moderate drought stress, SDS = severe drought stress, FT = foliar treatments, WS = water spray, MLE-LM = moringa leaf extract from local landrace of Multan origin, LF = local landrace of Faisalabad origin, LD = local landrace of DG Khan origin, EL = exotic landrace, WT = water treatments

**Table 3:** Impact of leaf extracts from local and exotic moringa landraces on number of kernels per panicle, 1000-kernal weight and grain yield of rice cultivated under different levels of drought stress (n = 4).

Treatments	Kernels per panicle				1000-kernel weight (g)				Grain yield (g)			
	CC	MDS	SDS	Mean (FT)	CC	MDS	SDS	Mean (FT)	CC	MDS	SDS	Mean (FT)
WS	104.75	90.50	70.50	88.58 D	24.64 ef	23.73 g	16.34 l	21.56 E	65.35	35.38	19.25	39.99 D
MLE-LM	114.75	96.00	76.25	95.67 B	25.93 b	24.97 de	20.18 i	23.68 B	71.25	50.75	27.25	49.75 B
MLE-LF	119.50	101.50	81.00	100.67 A	28.07 a	26.11 b	21.37 h	25.18 A	75.50	55.50	30.00	53.67 A
MLE-LD	113.75	96.50	76.50	95.58 B	25.68 bc	24.98 de	19.40 j	23.35 C	70.50	52.00	25.99	49.49 B
MLE-EL	111.50	94.00	73.00	92.83 C	25.24 cd	24.18 fg	18.34 k	22.58 D	69.50	45.50	24.25	46.42 C
Mean (WT)	113.00 A	96.00 B	76.00 C		25.91 A	24.79 B	19.12 C		70.42 A	47.82 B	25.34 C	
LSD, 0.05	WT = 0.8535, FT = 1.1636, WT×FT = NS				WT = 0.2090, FT = 0.3235, WT×FT = 0.5603				WT = 0.7855, FT = 0.8574, WT×FT = NS			

Means sharing the same alphabets did not differ significantly at P ≤ 0.05. NS = statistically non-significant, CC = control condition, MDS = moderate drought stress, SDS = severe drought stress, FT = foliar treatments, WS = water spray, MLE-LM = moringa leaf extract from local landrace of Multan origin, LF = local landrace of Faisalabad origin, LD = local landrace of DG Khan origin, EL = exotic landrace, WT = water treatments

The highest amylose contents (%) in rice kernels were recorded under CC followed by MDS, SDS resulted in the lowest amylose content (Table 4). Among MLE from various landraces, MLE-LF recorded the highest amylose contents followed by MLE-LM, MLE-LD and MLE-EL, respectively (Table 4). Amylopectin contents (%) were significantly altered by drought stress and MLE treatments. The highest and the lowest amylopectin contents (%) were recorded for WS and MLE-LF, respectively. Similarly, MLE from other landraces also noted lower amylopectin contents (%) than WS (Table 4). Protein contents (%) were altered by drought stress treatments; however, MLE and interactive effect of drought stress and MLE treatments were non-significant. The highest protein contents were observed under SDS followed by MDS, whereas CC recorded the lowest protein contents (Table 4).

The article "Moringa leaf extract improves biochemical attributes, yield and grain quality of rice (Oryza sativa L.) under drought stress" was retracted in 2022. Reasons: compromised peer review; a conflict of interest; concerns about the authorship.

**Table 4:** Impact of leaf extracts from local and exotic moringa landraces on amylose, amylopectin and protein contents in rice grains cultivated under different levels of drought stress (n = 4).

Treatments	Amylose contents (%)				Amylopectin contents (%)				Protein contents (%)			
	CC	MDS	SDS	Mean (FT)	CC	MDS	SDS	Mean (FT)	CC	MDS	SDS	Mean (FT)
WS	23.20	20.20	16.45	19.95 D	76.80	79.80	83.55	80.05 A	6.22	7.60	10.20	8.01
MLE-LM	24.15	21.46	18.05	21.20 B	75.80	78.52	81.95	78.77 C	6.25	7.70	10.10	8.02
MLE-LF	24.70	22.15	19.70	22.18 A	75.30	77.85	80.30	77.82 D	6.05	7.27	10.12	7.82
MLE-LD	24.20	21.45	18.15	21.27 B	75.80	78.55	81.85	78.73 C	6.02	7.35	10.37	7.92
MLE-EL	23.70	20.75	17.25	20.57 C	76.30	79.25	82.75	79.43 B	6.10	7.45	10.32	7.96
Mean (WT)	23.99 A	21.21 B	17.92 C		76.01 C	78.79 B	82.08 A		6.13 C	7.46 B	10.22 A	
LSD, 0.05	WT = 0.0544, FT = 0.1087, WT×FT = NS				WT = 0.0445, FT = 0.4481, WT×FT = NS				WT = 0.1084, FT = NS, WT×FT = NS			

Means sharing the same alphabets did not differ significantly at *P ≤ 0*.*05*. NS = statistically non-significant, CC = control condition, MDS = moderate drought stress, SDS = severe drought stress, FT = foliar treatments, WS = water spray, MLE-LM = moringa leaf extract from local landrace of Multan origin, LF = local landrace of Faisalabad origin, LD = local landrace of DG Khan origin, EL = exotic landrace, WT = water treatments

## Discussion

The current study revealed that MLE application significantly improved gas exchange attributes, physiological responses, enzymatic activities and productivity of rice crop under drought stress. The findings relating to gas exchange attributes are in agreement with previous studies reporting that drought stress significantly reduced *A*, *gs* and *E* [28, 29]. The *A* and other activities in flag leaf are the major source of crop productivity; however, these are susceptible to abiotic stresses, including drought stress [30]. The current study indicated that *A*, *gs* and *E* were significantly decreased (Fig 1A–1C) under drought stress. Liu [31] concluded that drought stress decreased net *A* and *gs* in rice crop. The stomatal closure of leaves limits CO_2_ uptake, which reduced the source size. Moreover, leaf senescence might also be a constraint to dry matter conversion to panicle during milking stage [32, 33].

Disturbed physiological activities might be responsible for low grain yield. Drought stress is responsible for reduced photosynthetic pigments and carotenoids (Fig 2A–2D). Concentrations of these pigments was linearly reduced with increasing drought intensity. Chlorophyll contents were decreased under drought stress in this study. These results are in line with Swapna [34], who stated that chlorophyll contents and carotenoids were reduced under drought stress in rice. It is also reported that drought could damage chlorophyll contents. Higher chlorophyll contents were observed for stress-free environment compared to drought-stressed environments [35]. It is also reported that drought stress can significantly decrease chlorophyll contents and the reduction increases with increasing intensity of drought [36]. Chlorophyll and photosynthetic parameters can be used as indicators to judge the degree of drought stress [37]. Drought stress decreases photosynthetic rate, water contents and transpiration and increases stomatal resistance [38].

Foliar application of MLE significantly improved gas exchange traits and photosynthetic pigments under drought stress (Figs 1 and 2). Moringa leaves possess considerable concentration of particular plant pigments with proven antioxidant properties such as chlorophyll and carotenoids (xanthin, beta-carotene, alpha-carotene and lutein) [39]. Furthermore, moringa leaves have many macro-elements which improved concentration of chlorophyll *a* & *b* in rice. It is also reported that MLE may stimulate earlier formation of cytokinins; thus, avoiding premature leaf senescence and resulting in higher leaf area with more photosynthetic pigments [40]. Findings of current study are also in line with Khan [17] who reported that application of MLE significantly enhanced photosynthetic pigments in wheat grown under benign conditions. Nawaz [7] reported that foliar application of MLE increases chlorophyll *a* and *b* in wheat crop when applied at tillering and heading stages. Improved growth with fresh MLE can be attributed to the presence of different secondary metabolites and allelochemicals such as phenols, ascorbates and zeatin [13]. These findings are also supported by Khan [14] that leaf extract of moringa landrace from Faisalabad origin (MLE-LF) showed higher biostimulant potential that might be due to the presence of higher concentration of biostimulant elements, plant growth promoting substances, mineral nutrients and antioxidants.

The article "Moringa leaf extract improves biochemical attributes, yield and grain quality of rice (Oryza sativa L.) under drought stress" was retracted in 2022. Reasons: compromised peer review; a conflict of interest; concerns about the authorship.

Antioxidant defense system plays key roles in plants’ tolerance to stressful environments. Application of MLE enhanced the activities of enzymatic antioxidant particularly under drought stress. Activities of enzymatic antioxidants were increased with the onset of drought stress (Fig 3A–3D). Our results showed that improved activities of SOD, CAT and APX might be linked to induction of antioxidant responses that protect the plant from oxidative damage. According to Foyer and Noctor [41], the initiation of activities of enzymatic antioxidants is a natural adaptation to overcome oxidative stress in plants. The SOD has been accepted as the basis of defense in response to oxidative stress [42]. The overexpression of SOD has been considered as a vital anti-drought mechanism [43], if accompanied by enhanced H_2_O_2_ scavenging mechanisms. Hanafy [44] reported significant increase in the activities of enzymatic antioxidants (GR, SOD and APX) in drought stressed soybean. SOD and APX activities were also increased in canola (*Brassica napus* L.) under drought stress [45]. Application of MLE caused significant increase in SOD activities in soybean followed by GR and APX, respectively. Zaki and Rady [46] reported that application of MLE as seed soaking or foliar spray improved activities of enzymatic antioxidants such as glutathione reductase, SOD and APX in common bean (*Phaseolus vulgaris* L.) plants.

The present study depicted the influence of growing environment, especially drought stress on growth, productivity, grain yield and quality of rice crop. Increasing levels of drought stress has a direct influence on crop growth and yield attributes (Tables 2 and 3). This reduction in growth and productivity under limited water availability can be linked to reduced photosynthetic capacity and photosynthetic area of leaves [47]. Various drought conditions adversely affected the enzymatic activities which reduced the growth and yield attributes of tomato crop [48]. These results are in agreement with Mukamuhirwa [49] who concluded drought stress significantly reduced growth parameters of rice plants. Farooq [50] reported that drought stress decreases plant growth by influencing many biochemical and physiological processes, including respiration, photosynthesis, ion uptake, translation, nutrient assimilation and carbohydrates metabolism. Exogenous application of MLE from all landraces significantly improved growth and yield parameters even under drought stress. However, foliar spray of MLE from Faisalabad landrace resulted in the highest improvement in grain yield under well-watered and/or drought stress circumstances (Table 4). Barnabas [51] stated that drought stress significantly reduced grain weight because of less number of endosperm cells, reduced starch synthesis and restricted translocation of photosynthates from source to sink [52]. Farooq [53] also investigated that exogenous application of water extract of brassica improved the root and shoot lengths as well as biomass of wheat and chickpea.

The article "Moringa leaf extract improves biochemical attributes, yield and grain quality of rice (Oryza sativa L.) under drought stress" was retracted in 2022. Reasons: compromised peer review; a conflict of interest; concerns about the authorship.

Foliar application of MLE significantly enhanced the performance of rice plants under drought stress which is obvious from the improved number of kernals, kernel weight and grain yield. These findings are supported by previous studies of Basra [16], Yasmeen [54] and Khan [9, 17] who reported that MLE acts as an exogenous plant growth promoter because of the presence of ascorbate, phenols, zeatin, carotenoids, antioxidants, essential plant mineral nutrients and vitamins. It is suggested that application of MLE as exogenous foliar spray might have improved endogenous hormonal levels thereby resulting in improved plant growth [9, 17, 55]. Discovered cytokinin in MLE have a vital role in the promotion chlorophyll biosynthesis, cell division and cell elongation [56]. Drought stress adversely affected amylose, amylopectin contents and protein contents in grains and MLE improved these parameters (Table 4). These results are consistent with the findings of Mukamuhirwa [57], who stated that drought adversely affected amylose contents in grains. The amylose content varied between 14% and 25%, corresponding to intermediate amylose content [58]. Generally, cultivars with high and intermediate amylose content have a stable content across seasons [59].

The article "Moringa leaf extract improves biochemical attributes, yield and grain quality of rice (Oryza sativa L.) under drought stress" was retracted in 2022. Reasons: compromised peer review; a conflict of interest; concerns about the authorship.

## Conclusion

Gas exchange traits, photosynthetic pigments, enzymatic activities, growth, yield and quality attributes of rice plants were adversely affected by the imposition of water deficit conditions as compared to well-watered environment. Foliar application of leaf extracts from all landraces significantly improved the gas exchange traits, photosynthetic pigments, enzymatic activities, growth, yield and quality traits under normal and water deficit conditions. However, MLE from Faisalabad landrace showed maximum biostimulant potential regarding improved gas exchange traits, higher photosynthetic pigments and maximum enzymatic activities of rice plants grown under normal as well as water deficit circumstances. It is concluded from the outcomes of current experimentation that the application of moringa leaf extract from Faisalabad landrace can be used to enhance the productivity of field crops under normal and water deficit conditions.
